The article "MiRNA-506 inhibits rheumatoid arthritis fibroblast-like synoviocytes proliferation and induces apoptosis by targetting TLR4" was retracted in 2021. Reasons: signs of a paper mill; concerns about the images.

# MiRNA-506 inhibits rheumatoid arthritis fibroblast-like synoviocytes proliferation and induces apoptosis by targetting TLR4

**DOI:** 10.1042/BSR20182500

**Published:** 2019-05-07

**Authors:** Dan Li, Qingchen Zhou, Gaojian Hu, Gang Wang

**Affiliations:** 1 Department of Radiology, The First Hospital of Jilin University, Changchun, Jilin 130021, P.R. China; 2 Department of Orthopedics, The Third Hospital of Jilin University, Changchun, Jilin 130033, P.R. China

**Keywords:** fibroblast-like synoviocytes, miR-506, Rheumatoid arthritis, TLR4

## Abstract

Fibroblast-like synoviocytes (FLSs) play a crucial role in rheumatoid arthritis (RA) pathogenesis. While miRNA (miR)-506 has been implicated in the progression of multiple diseases, its role in RA remains to be explored. The present study evaluated the function of miR-506 in the regulation of RA-FLSs. FLSs were prepared from RA and healthy synovial tissues. The expression of miR-506 was measured by quantitative real time PCR (qRT-PCR). The effects of miR-506 on RA-FLSs proliferation and apoptosis were detected by cell counting Kit-8 and flow cytometry assays, respectively. The determination of TNF-α, IL-6, and IL-1β concentrations in RA-FLSs supernatant were done by ELISA. The levels of miR-506 were detected to be significantly lower in the synovial tissues and FLSs of RA than in the synovial tissues and FLSs of healthy controls. The miR-506 up-regulation in RA-FLSs significantly inhibited the proliferation and promoted cell cycle arrest at the G_0_/G_1_ phase. The overexpression of miR-506 induced apoptosis, along with an increase in activities of caspase-3 and -8. A target gene *Toll-like receptor 4* (*TLR4*) under the direct regulation of miR-506 was identified through the luciferase assay, qRT-PCR and western blot analysis. Forced overexpression of *TLR4* in the rescue experiments showed that TLR4 effectively reversed the effect on proliferation and apoptosis in miR-506-overexpressing RA-FLSs. Thus, miR-506 may be a potential target for RA prevention and therapy of RA.

## Introduction

As a chronic and systemic inflammatory disease, rheumatoid arthritis (RA) is identified through symptoms such as hyperplasia of the synovium and extraarticular manifestations, which leads to cartilage damage, joint destruction, and deformation [1]. In the pathogenesis of RA, a key role is played by the fibroblast-like synoviocytes (FLS) within the synovial intimal lining [2]. RA-FLSs are similar to malignant cancer cells in some properties, such as resistance to apoptosis, uncontrolled growth, and high invasiveness [3]. Thus, to explore therapeutic strategies to treat RA, it is urgent need to find molecular mechanisms of the aggressive phenotype of RA-FLSs.

The article "MiRNA-506 inhibits rheumatoid arthritis fibroblast-like synoviocytes proliferation and induces apoptosis by targetting TLR4" was retracted in 2021. Reasons: signs of a paper mill; concerns about the images.

In recent years, studies on small non-coding RNAs (miRNAs) have widely focussed on multiple diseases because of their involvement in the regulation of several physiological and pathological processes, including cell metabolism, proliferation, migration, invasion, and inflammation [4,5]. Abnormal miRNAs have been reported to be associated with the occurrence and development of RA, suggesting miRNAs as a diagnostic marker or therapy target of RA [6,7].

The role of miR-506 as a tumor suppressor or oncogene has been widely studied in different cancers [8–15]. A recent study showed that miR-506 could regulate the NFκB signal pathway in osteosarcoma [11]. However, the functional significance and molecular mechanisms underlying the role of miR-506 in RA remain unclear. Therefore, we undertook the present study to examine the effect of miR-506 in healthy and RA synovial tissues and in FLSs; to evaluate the effects of miR-506 on RA-FLS proliferation, cell cycle arrest, apoptosis, and inflammatory cytokines; and to explore the mode of miR-506 action in RA-FLSs.

## Materials and methods

### Samples of tissues

A total of 24 patients of RA (12 men and 12 women; mean age, 55.4 ± 7.2 years) took part in the study, and their synovial tissues were obtained during knee replacement surgery. The diagnosis of RA was done as per 2010 classification criteria for RA defined by the American College of Rheumatology/European League against Rheumatism [16]. Healthy synovial tissues from 12 patients (six men and women each; mean age, 44.4 ± 6.3 years) with a traumatic knee condition were collected and used as normal control. Informed consent was obtained from all the patients. The study protocol was reviewed and approved by the Ethics Committee of The First of Hospital, Jilin University. The study was undertaken in accordance with the ethical standards of the World Medical Association Declaration of Helsinki.

### Assays using cell culture and transfection

Normal human FLSs and RA-FLSs were brought from Cell Applications (San Diego, CA, U.S.A.). For cell-culture, DMEM (Invitrogen, Carlsbad, CA, U.S.A.) was used and augmented with FBS (10%; HyClone, UT, U.S.A.), 100 units/ml penicillin or 100 μg/ml streptomycin. The cells were grown at 37°C in an atmosphere with appropriate humidity, and 5% CO2. MiR-506 mimic and oligonucleotide negative control (miR-NC) were brought from the GenePharm (Shanghai, China) and transfected into the RA-FLSs cells by using Lipofectamine 2000 (Invitrogen, CA, U.S.A.) as per instructions of the manufacturer.

### Isolation of RNA and qRT–PCR

The cultured FLSs and tissue samples were used for miRNA extraction using the miRNA Isolation Kit mirVana supplied by Ambion (Carlsbad, CA, U.S.A.) as per protocol defined by the manufacturer. For the distinct quantitation of miR-506 expression, TaqMan miRNA assays (Applied Biosystems, Carlsbad, CA, U.S.A.) with specific primers and probes were done as per instructions specified by the manufacturer. To detect the expression level of *TLR4* mRNA, TRIzol reagent (Invitrogen) was used to extract total RNA from tissues or RA-FLSs and reverse transcribed to cDNA using the Primer Script RT reagent Kit from TaKaRa (Dalian, Japan). For the qPCR assay, Fast SYBR Green Master Mix from Applied Biosystems (CA, U.S.A.) along with the GAPDH and TLR4 primers were used and carried out on the ABI-7900HT machine (Applied Biosystems), as reported previously [17]. U6 and GAPDH were applied as internal controls for miR-506 and TLR4 mRNA. The relative expression miR-506 and TLR4 were calculated with the using the 2^–∆∆*C*^_T_ method.

The article "MiRNA-506 inhibits rheumatoid arthritis fibroblast-like synoviocytes proliferation and induces apoptosis by targetting TLR4" was retracted in 2021. Reasons: signs of a paper mill; concerns about the images.

### Determination of protein concentration

FLSs transfected with either miR-506 or miR-NC were cultured for 24 h. Then, TNF-α, IL-1β, and IL-6 concentrations in the cell culture supernatant were assessed by ELISA according to kit instructions.

### Cell proliferation

For the RA-FLSs proliferation assay, Cell Counting Kit-8 (CCK-8; Dojindo, Kumamoto, Japan) was used. Concisely, in a 96-well plate, the transfected RA-FLSs were seeded at 1 × 10^4^ cells/well and grown at 37˚C in an incubator for 24–72 h in 5% CO2. The cell viability was evaluated at specified time points (24, 48, and 72 h) using the CCK-8 kit as per instructions of the manufacturer. The detection of absorbance (450 nm) per well was done using a microtiter plate reader from Molecular Devices (CA, U.S.A.).

### Determination of cell cycle distribution and apoptosis through flow-cytometry

For cell cycle distribution assay, the RA-FLS transfected with miR-506 or miR-NC were fixed using ethanol (70%) and kept at 4°C for 15 min in a staining solution with RNase A (200 μg/ml) and PI (propidium iodide; 50 μg/ml; Sigma–Aldrich). The analysis of cell arrest was done using a FACSCalibur flow cytometer from Beckman Coulter (Fullerton, CA, U.S.A.). The Apoptosis Detection Kit Annexin V-FITC procured from eBioscience (San Diego, CA, U.S.A.) was used to determine cell apoptosis, which was then quantitated flow cytometrically (FACSort; Becton) as per instructions of the manufacturer.

### Assay for caspase-3 and -8 activities

After 48 h of RA-FLSs transfection, activities of caspase-3 and -8 were carried out using a colorimetric assay kit from BioVision (CA, U.S.A.) as per instructions of the manufacturer. Finally, absorbance (405 nm) was measured using a microtiter plate reader from Molecular Devices.

The article "MiRNA-506 inhibits rheumatoid arthritis fibroblast-like synoviocytes proliferation and induces apoptosis by targetting TLR4" was retracted in 2021. Reasons: signs of a paper mill; concerns about the images.

### Luciferase reporter assay

To predict target genes of miR-506, three publicly available algorithms: TargetScan, PicTar, and miRBase were used. TLR4 was chosen as a target of miR-506. The 3′-UTR regions of *TLR4* with the putative binding- (WT) or mutant-sites (MT) for miR-506 were synthesized by GenePharm (Shanghai, China). These oligonucleotides were cloned in the pGL3 vector procured from Ambion (Austin, TX, U.S.A.), and were labeled as WT-TLR4-3′ UTR, and MT-TLR4-3′ UTR. For the luciferase reporter assay, RA-FLSs were cotransfected with miR-506 mimic or miR–NC and reporter plasmids WT-TLR4 -3′ UTR or MT-TLR4-3′ UTR along with Lipofectamine 2000. After transfecting for 48 h, activities of Renilla and firefly luciferase were determined using a Dual-Luciferase^®^ Reporter assay kit procured from Promega (Madison, U.S.A.) as per the method defined by the manufacturer. The results are presented as the ratio of firefly: Renilla luciferase activities.

### Determination of protein levels

A RIPA (radioimmunoprecipitation) lysis buffer from Beyotime (Shanghai, China) was used to isolate total proteins from cultured RA-FLSs. The determination of the concentration of total protein was carried out employing a BCA protein assay kit procured from Pierce (Rockford, IL, U.S.A.). Proteins in equal, and measured amounts were electrophoretically separated on SDS-PAGE (10%) and transferred to PVDF membranes (polyvinylidene fluoride; Millipore, U.S.A.). After the blocking procedure with nonfat milk (5%), antibodies against TLR4 (1:2000), CyclinA1(1:1000), CyclinB1(1:1000), CyclinD2(1:2000), and GAPDH (1:5000) (all from Santa Cruz, U.S.A.) were added to the membrane, followed by secondary antibodies (1:6000, Santa Cruz) conjugated with horseradish peroxidase. The internal loading control was GAPDH. The chemiluminescent substrate kit from Millipore Company (Bedford, MA, U.S.A.) was used to observe protein bands as per instructions of the manufacturer. Gray analysis was performed using software Gel-Pro Analyzer 4 (United States Biochemical, Cleveland, OH, U.S.A.).

### Statistical analyses

For each analysis, experiments were done independently thrice and the outcomes are mentioned as the mean ± S.D. The (two-tailed) Student’s *t*-test was applied for quantitatively comparing the data between two groups and significant values were *P*<0.05. Between three or more groups, one-way ANOVA along with Bonferroni *post hoc* tests were carried out and a significant value was *P*<0.05. The relationship between the expressions of miR-506 and *TLR4* mRNA was evaluated by Spearman’s correlation coefficient. For all analysis, the SPSS 19 software from SPSS Inc (Chicago, IL, U.S.A.) was used.

The article "MiRNA-506 inhibits rheumatoid arthritis fibroblast-like synoviocytes proliferation and induces apoptosis by targetting TLR4" was retracted in 2021. Reasons: signs of a paper mill; concerns about the images.

## Results

### Down-regulation of miR-506 in RA synovial tissues and FLSs

The qRT-PCR was carried out to measure the expression of miR-506 in synovial tissues from RA patients and healthy controls. The levels of miR-506 in RA-affected synovial tissues were lower compared with that in the healthy controls (Figure 1A). Consistently, miR-506 expression was significantly decreased in human RA-FLSs compared with normal human FLSs (*P*<0.05; Figure 1B). Thus, an alteration miR-506 expression may be possibly associated with the RA pathogenesis.

**Figure 1:** miR-506 expression level is down-regulated in RA synovial tissues and FLSs (**A**) The relative expression of miR-506 in synovial tissue from RA patients (*n*=24) or healthy control (normal, n = 12) was examined by qRT-PCR. (**B**) The relative expression of miR-506 in FLSs from RA patients (RA-FLSs) or healthy control (normal-FLSs) was examined by qRT-PCR. **, *P*<0.01 vs. Normal-synovial and Normal-FLSs groups.

### Up-regulation of miR-506 suppresses the proliferation of RA-FLSs

We used miR-506 mimic to transfect RA-FLSs to restore the expression of miR-506 and to assess its function in RA and confirmed the same through qRT-PCR. The RA-FLSs transfected with miR-506 mimic showed a 5.4-fold increase in miR-506 expression (Figure 2A). We also observed through CCK-8 assay that the proliferation of RA-FLSs was significantly inhibited due to overexpression of miR-506 (Figure 2B). Since the proliferation of cell and the cell cycle distribution are closely connected, we also evaluated the result of miR-506 on the arrest of cell cycle. Flow cytometric analysis revealed that miR-506 overexpressed in RA-FLSs led to significant increase in the G_1_/G_0_-phase cells (79.5 ± 7.4% vs 62.6 ± 5.5%) and a decrease in the of S-phase cells (11.2 ± 1.1% vs 28.4 ± 1.6%), compared with that in RA-FLSs transfected with miR-NC (Figure 2C). Moreover, several cell cycle factors (Cyclin A1, CyclinB1, and CyclinD2) were determined by western blot. The results demonstrated that miR-506 overexpression significantly decreased Cyclin A1, Cyclin B1, and CyclinD2 protein expression in RA-FLSs. These results suggested that miR-506 miR-506 overexpression inhibits cell proliferation by regulating cell cycle arrest in RA-FLSs.

**Figure 2:** Up-regulation of miR-506 suppresses the proliferation of RA-FLSs (**A**) miR-506 expression levels were determined in RA-FLSs transfected with miR-506 mimic or miR-NC mimic by qRT-PCR. (**B**,** C**) Cell proliferation and cell cycle arrest were determined in RA-FLSs transfected with miR-506 mimic or miR-NC. (**D**) The Cyclin A1, CyclinB1, and CyclinD2 proteins expression were determined in RA-FLSs transfected with miR-506 mimic or miR-NC by western blot. GAPDH was used to as internal control. *, *P*<0.05; **, *P*<0.01 vs. miR-NC group.

The article "MiRNA-506 inhibits rheumatoid arthritis fibroblast-like synoviocytes proliferation and induces apoptosis by targetting TLR4" was retracted in 2021. Reasons: signs of a paper mill; concerns about the images.

### Up-regulation of miR-506 promotes the apoptosis of RA-FLSs

Next, we carried out flow-cytometry to evaluate the extent to which miR-506 affects RA-FLSs apoptosis and observed that overexpression of miR-506 in RA-FLSs significantly increase apoptosis ratio in contrast with RA-FLSs transfected with miR-NC (19.9 ± 1.62% vs 5.3 ± 0.8%, *P*<0.05; Figure 3A). Additionally, the activities of caspase-3 and -8 significantly increased in miR-506 overexpressing RA-FLSs (Figure 3B,C). Thus, these results suggested that miR-506 could trigger apoptosis of RA-FLSs.

**Figure 3:** Up-regulation of miR-506 promotes the apoptosis of RA-FLSs (**A**) Cell apoptosis was detected in RA-FLSs transfected with miR-506 mimic or miR-NC mimic by flow cytometric analysis. (**B**,** C**) The activities of caspase-3 and -8 were determined in RA-FLSs transfected with miR-506 mimic or miR-NC mimic by ELESA. *, P<0.05; **, *P*<0.01 vs.miR-NC group.

### Up-regulation of miR-506 suppresses inflammatory cytokines release of RA-FLSs

To assess the role of miR-506 on the inflammatory cytokines secreted by RA-FLSs, we determined the TNF-α, IL-6, and IL-1β levels in RA-FLSs transfected with miR-506 mimic or miR-NC. The ELISA assay demonstrates that miR-506 overexpression drastically impeded the IL-1β, IL-6, and TNF-α release (Figure 4A-C), suggesting that miR-506 might suppress the secretion of inflammatory cytokines in RA-FLSs.

**Figure 4:** Up-regulation of miR-506 suppresses inflammatory cytokines release of RA-FLSs (**A-C**) RA-FLS transfected with miR-506 mimic significantly reduced production of TNF-a(A), IL-1β(B), and IL-6(C) compared with RA-FLSs transfected with miR-NC. **, *P*<0.01 vs. miR-NC group.

### miR-506 acts directly on TLR4 in RA-FLSs

MiRNAs implicated in various roles by regulating target genes [4]. Thus, to identify potential target genes that could be regulated by miR-506 in RA-FLSs, the PicTar, TargetScan, and miRanda bioinformatic databases were used, and based on a binding sequence at 300–306 bp of *TLR4* 3′-UTR, a potential target for miR-506 was selected (Figure 5A). To explore whether miR-506 targets *TLR4*, RA-FLSs were co-transfected with the plasmid containing luciferase reporter with either mutant-type (MT) or wild-type (WT) *TLR4*, and miR-506 mimic or miR-NC and 48 h after transfection, luciferase activity in these cells was estimated. As shown in Figure 5B, the activity of luciferase in cells transfected with *TLR4*- WT and miR-506 was remarkably reduced when compared with that of the miR-NC with *TLR4*-WT group as well as that of miR-506 with *TLR*-MUT, respectively. Moreover, overexpression of miR-506 decreased TLR4 expression on both the mRNA and protein levels (Figure 5C,D), while an increased *TLR4* expression was observed in RA synovial tissues (Figure 5E), and its expression correlated inversely with that of miR-506 in RA synovial tissues (Figure 5F). These results imply that *TLR4* might be a target of miR-506 in RA-FLSs.

The article "MiRNA-506 inhibits rheumatoid arthritis fibroblast-like synoviocytes proliferation and induces apoptosis by targetting TLR4" was retracted in 2021. Reasons: signs of a paper mill; concerns about the images.

**Figure 5:** TLR4 is a direct target of miR-506 in RA-FLSs (**A**) Sequence alignment of WT and MT putative miR-506-binding sites in the 3′-UTR of TLR4 were shown. (**B**) Relative luciferase activity was detected in RA-FLSs co-transfected with WT or MT 3ʹ-UTR TLR4 reporter plasmids and miR-506 mimic or miR-NC. (**C, D**) TLR4 expression on mRNA and protein levels was examined in RA-FLS RA-FLSs transfected with miR-506 mimic or miR-NC mimic. GAPDH was used as an internal control. (**E**) Relative *TLR4* mRNA expression was detected in synovial tissues from RA patients and health donor. GAPDH was used as an internal control. (**F**) The correlations between *TRL4* mRNA expression level and miR-506 were analyzed in human synovial tissues by spearman’s correlation analysis. *, *P*<0.05; **, *P*<0.01 vs. miR-NC group.

### TLR4 overexpression reverses the impact of miR-506 on the proliferation and apoptosis of RA-FLSs

To assess whether miR-506 exerts biological function by regulating TLR4, we co-transfected RA-FLSs with miR-506 mimic and the TLR4 overexpression plasmid (lack of 3′-UTR). We found that miR-506-mediated TLR4 down-regulation was restored following co-transfection (Figure 6A). Furthermore, forced expression of TLR4 also reversed the effect of miR-506 in RA-FLSs proliferation, cycle arrest, and apoptosis (Figure 6B–D). Thus, miR-506 may exert a suppressive role in RA-FLSs by repressing TLR4.

**Figure 6:** The impact of miR-506 on the proliferation and apoptosis of RA-FLSs was reversed by TLR4 overexpression (**A**) TLR4 protein expression was determined in RA-FLSs transfected with miR-506 mimic or miR-NC and with/without TLR4 overexpression vector (lack of 3′-UTR). GAPDH was used as an internal control. (**B–D**) The effect of miR-506 on cell proliferation, cycle arrest, and apoptosis in RA-FLSs was reversed under the condition of overexpression of TLR4. *, *P*<0.05; **, *P*<0.01 vs. miR-NC group.

## Discussion

Accumulating evidence suggests that altered expression miRNAs might be involved in modulating the RA-associated inflammatory innate immune responses via the regulation of target genes [6,7]. For example, Gao et al. showed that miR-126 significantly promote growth and resistance to apoptosis in RA-FLS by targetting PIK3R2 and indirectly regulating PI3K/AKT signaling pathway [18]. Li et al reported that when miR-192 was expressed ectopically, it led to a remarkable increase in the arrest of the cell cycle at G_0_/G_1_ phase, inhibition of proliferation, and repressed caveolin 1 (CAV1) which promoted activities of caspase-3 and -8 in RA-FLSs [19]. Liu et al reported that miR-29a overexpression in RA-FLS remarkably promoted apoptosis, inhibited proliferation, and repressed inflammatory cytokine expression by targetting STAT3 (signal transducer and activator of transcription 3) [20]. In the current study, we found that the expression of miR-506 was markedly down-regulated in synovial tissues and FLS of RA patients compared with health donor. To determine its function in the RA-FLSs pathophysiology, we also investigated how miR-506 affects cell proliferation and apoptosis and found that restoration of miR-506 notably suppressed cellular proliferation and induced apoptosis in RA-FLSs; thus, strongly indicating that miR-506 might have a key role in RA progression.

The article "MiRNA-506 inhibits rheumatoid arthritis fibroblast-like synoviocytes proliferation and induces apoptosis by targetting TLR4" was retracted in 2021. Reasons: signs of a paper mill; concerns about the images.

It has been documented that miR-506 exerts growth inhibitory effects on many types of cancers, such as colorectal cancer [10], neuroblastoma [18], pancreatic cancer [9], osteosarcoma [11], glioma [12], breast cancer [14], and cervical cancer [15]. However, in colon cancer [21] and melanoma [22], miR-506 functioned as an oncogene. The contrasting effects miR-506 exerts on different types of cancer cell lines indicate that miR-506 might perform different roles dependent on different cell types. The results of the present study were extended to nonmalignant cells and showed that miR-506 overexpression remarkably repressed RA-FLSs proliferation, and arrested them at the G_0_/G_1_ phase. We also showed that miR-506 overexpression significantly induced apoptosis and increased the activities of caspase-3 and -8 in RA-FLSs, and reduced the secretion of inflammatory cytokines in RA-FLSs. Therefore, miR-506 plays an inhibitory role in the development of RA-FLSs.

It was well known that miRNAs exerts its biological roles by regulating target genes [4]. Thus, to further understand the underlying mechanisms by which miR-506 inhibits the growth of RA-FLSs, we sought to identify its direct target genes. Three algorithms (TargetScan, miRanda, and miRDB) were used to predict candidate target of miR-506. Amongst target genes, TLR4 was selected for further investigation based on its biological functions. Accordingly, luciferase reporter assay showed that miR-506 could specifically bind with the 3′-UTR of TLR4. In addition, overexpression of miR-506 significantly decreased TLR4 expression on mRNA and protein levels in RA-FLSs. These data suggested that TLR4 was a direct target of miR-506 in RA-FLSs. TLR4 has been reported to play a key role in RA pathogenesis by regulating the production of inflammatory cytokines [23,24]. Recently, studies showed that TLR4 expression was up-regulated in synovial tissues and RA-FLSs [25], and that TLR4 promotes pathological progression of RA by increasing the secretion of matrix metalloproteinase3 as well as IL-6 and IL-8 in RA-FLSs [26]. Importantly, TLR4 could regulate several miRNAs in RA-FLS, including miR-140-5p [24], miR-146a [27], miR-548a-3p [28], miR-27a [29], and miR-20a [30]. In agreement, we showed that TLR4 mRNA expression levels were up-regulated in synovial tissues, and its expression level was negative correlated with miR-506. Of note, the effects of miR-506 on proliferation and apoptosis in RA-FLSs were reversed by overexpression of TLR4. These results suggested that miR-506 exerted it inhibitory function in RA-FLSs, at least in part, by targetting TLR4.

The article "MiRNA-506 inhibits rheumatoid arthritis fibroblast-like synoviocytes proliferation and induces apoptosis by targetting TLR4" was retracted in 2021. Reasons: signs of a paper mill; concerns about the images.

There were several limitations in our experiment. First, the biological function of miR-506 was evaluated through up-regulation of miR-506 in an RA-FLS gain-of-function model. Concurrently, loss-of-function studies through the down-regulation of miR-506 in RA-FLSs are required to further verify our findings. Second, The RA sample-size was limited, and more samples need to be investigated for the clinical significance of miR-506. Third, the miR-506 may be involved in RA progression through multiple target genes, and the underlying molecular mechanisms must be analyzed in the future.

To summarize, this is the first study to assess the role of miR-506 on human RA-FLSs. While the miR-506 is repressed in RA synovial tissues and FLSs, miR-506 overexpression inhibits cell proliferation by regulating cell cycle arrest, promotes apoptosis and caspase-3 and -8 activities, as well as decreases the secretion of inflammatory cytokines in RA-FLSs by targetting TLR4. Thus, miR-506 might be a promising candidate for therapies involving prevention of RA progression.

## Abbreviations

CCK-8: cell counting kit-8
FLS: fibroblast-like synoviocyte
MT: mutant type
PI: propidium iodide
qRT-PCR: quantitative real time PCR
RA: rheumatoid arthritis
TLR4: Toll-like receptor 4
WT: wild type
